# Comparison of Clinical Efficacy and Safety between Misoprostol and Oxytocin in the Prevention of Postpartum Hemorrhage: A Meta-Analysis

**DOI:** 10.1155/2022/3254586

**Published:** 2022-04-11

**Authors:** Renmei Xu, Yongjie Guo, Qinggui Zhang, Xiaokang Zeng

**Affiliations:** ^1^Department of Intensive Care Unit, Jiaxing Maternity and Child Health Care Hospital, Jiaxing 314000, China; ^2^Department of Intensive Care Unit, Affiliated Hangzhou First People's Hospital, Zhejiang University School of Medicine, Hangzhou 310006, China

## Abstract

In order to systematically evaluate the clinical efficacy and safety of misoprostol versus oxytocin in the prevention of postpartum hemorrhage, this paper provides evidence-based reference for clinical medication, computerized retrieval of Chinese biomedical literature database (CBM), PubMed, Embase, Cochrane Library, and clinical trials. The retrieval period is from the establishment of each database to October 1, 2021. Published randomized controlled trials (RCTS) are included in this study. The literature is screened and evaluated according to inclusion and exclusion criteria, and meta-analysis is performed using RevMan 5.3 software. A total of 13 RCTS are included, with a total of 24754 parturients. The meta-analysis shows the average blood loss (SMD = 0.10, 95% CI (−0.11, 0.32), *P*=0.35), the time of the third stage of labor (SMD = 0, 95% CI (−0.07, 0.08), *P*=0.95), and blood transfusion rate (RR = 0.80, 95% CI (0.63, 1.02), *P*=0.07). However, the incidences of shivering (RR = 2.61, 95% CI (1.79, 0.81), *P* < 0.00001) and vomiting (RR = 2.78, 95% CI (1.85, 4.18), *P* < 0.00001) are significantly higher than those in oxytocin group. The effect of misoprostol on preventing postpartum hemorrhage is similar to that of oxytocin, but the incidence of adverse reactions is high, and the occurrence of adverse reactions should be closely watched in the use process. Due to the limitations of the included studies, multicenter, large-sample, and high-quality RCTS are still needed in the future to further verify this conclusion.

## 1. Introduction

Postpartum hemorrhage is the main cause of maternal death and remains an urgent problem to be solved [1]. Related studies show that maternal deaths due to postpartum hemorrhage account for 80% of the total number of maternal deaths, and the important cause of postpartum hemorrhage is uterine contraction weakness [2]. In recent years, with the continuous development of obstetric medical technology, although the mortality rate of maternal direct death from postpartum hemorrhage is decreasing year by year, postpartum hemorrhage is still the first cause of maternal death [3, 4].

In order to avoid postpartum hemorrhage as far as possible, reasonable and effective preventive measures should be formulated early in clinical practice, followed by timely drug prevention intervention combined with the actual situation of parturients, so as to effectively reduce the amount of maternal bleeding and reduce mortality. The World Health Organization (WHO) recommends intramuscular injection of oxytocin as a standard preventive measure for postpartum hemorrhage [5]. However, oxytocin needs to be stored in cold storage and administered by injection, making it difficult to use in underdeveloped countries or remote areas. Misoprostol is an analogue of prostaglandin E1, which has a strong uterine contraction effect. In addition, misoprostol is cheap, does not need refrigeration, and can be administered orally [6]. Therefore, misoprostol can be considered as a drug to prevent postpartum hemorrhage in underdeveloped countries or remote areas. In recent years, a number of multicenter double-blind trials have been conducted to study the effect of misoprostol on the prevention of postpartum hemorrhage, but various studies have reported different results on the efficacy and safety of misoprostol, and the conclusions obtained are of limited reference value [7–9].

In view of the fact that there is no more use of misoprostol and oxytocin alone to prevent postpartum hemorrhage the clinical curative effect and security of the system evaluation or meta-analysis, in order to further clear the clinical value of misoprostol alone, this research adopts the meta-analysis method, system evaluation, with misoprostol compared efficacy and safety of the oxytocin alone to prevent postpartum hemorrhage in order to provide evidence-based evidence for evaluating whether misoprostol alone can be used as a substitute for oxytocin in the prevention of postpartum hemorrhage in underdeveloped countries or remote areas.

## 2. Inclusion and Exclusion Criteria

Inclusion criteria: (1) published randomized controlled trials (RCTS) are included in this study, regardless of whether blind method is adopted or not, without limitation of region or language; (2) the subjects of this study are women who delivered vaginal delivery or cesarean section, and their race, nationality, age, gestational age, gestational rank, and so on are not limited; (3) women in the experimental group are given misoprostol orally or sublingual, and women in the control group are given oxytocin intramuscular injection. The dosage of the two groups is not limited; (4) outcome indicators: the outcome indicators of this study included (1) average blood loss; (2) time of the third stage of labor; (3) blood transfusion rate; (4) incidence of shivering; and (5) incidence of vomiting. The exclusion criteria of this study included (1) summary of experience, case report, summary, letter, summary of meeting, and too little or incomplete information; (2) studies with fewer than 50 cases; (3) studies in which the route of administration of misoprostol is anus.

### 2.1. Search Strategy

Computerized retrieval of Chinese biomedical literature database (CBM), PubMed, Embase, Cochrane Library, and clinical trials: the retrieval period is from the establishment of each database to October 1, 2021. The mesh terms of misoprostol oxytocin postpartum hemorrhage were used for search, and we manually retrieved the included literature references.

### 2.2. Data Extraction and Quality Evaluation

Basic data (first author, year of publication, country of study, number of cases, age, and intervention) and outcome indicators (mean blood loss, time to the third stage of labor, blood transfusion rate, incidence of chills, and incidence of vomiting) are independently screened and extracted by 2 investigators. In the extraction process, if there is any difference of opinion, the third researcher will participate in the discussion and decide. If the outcome index data of the relevant study is unclear or missing, the researcher should contact the corresponding author of the literature as much as possible to obtain accurate original data and exclude the literature that cannot obtain data or information.

Cochrane Bias Risk Assessment Tool 5.3.0 is used to evaluate the quality of the included literature, including the random sequences generation, allocation concealment, blinding of participants and personnel, blinding of outcome assessment, incomplete outcome data, selective reporting, and other biases. Each item is assessed as low risk, unclear risk, and high risk of bias [10].

## 3. Statistical Method

Meta-analysis is performed using RevMan 5.3 software. Standard mean difference (SMD) is used as the effect analysis statistic for continuous variables, relative risk (RR) is used as the effect analysis statistic for classification variables, and 95% confidence interval (CI) is used for interval estimation. *χ*^2^ test is used to test the heterogeneity of the included studies. If there is no statistical heterogeneity among the results (*P* > 0.10, I2 ≤ 5%), fixed-effect model is used for meta-analysis. Otherwise, random-effects model is used for meta-analysis. At the same time, the source of heterogeneity is analyzed, and the possible heterogeneity factors are subgroup analyzed. In sensitivity analysis, the same index is repeatedly analyzed, and one study is gradually deleted to show the influence of one study on the merger effect, and then the influence of the study on the index is excluded. An inverted funnel plot is drawn for publication bias analysis.

## 4. The Experimental Result

### 4.1. Literature Screening and Basic Information of Included Literature

A total of 844 related articles are obtained in the preliminary searching. After further reading, 13 RCTS are finally included, with a total of 24754 pregnant women, including 12,372 cases in the experimental group (misoprostol group) and 12,382 cases in the control group (oxytocin group) [11–15]. The literature screening process is shown in Figure 1, and the basic information of the included literature is shown in Table 1.

### 4.2. Risk of Bias in Included Studies

All the studies described the specific random sequence generation methods and reported the allocation of hidden, blind methods; data are complete. Except for Chaudhuri, 2012, Elbohoty, 2016, and Bellad, 2012, which show that there are no other sources of bias in the results of selective reporting, all the other studies did not clearly indicate the results of selective reporting and whether there are other sources of bias.  Figure 2 presents risk of bias summary and risk of bias graph.

## 5. Results of Meta-Analysis and Sensitivity Analysis

### 5.1. Mean Blood Loss

Seven studies (2724 women) reported mean blood loss, with statistical heterogeneity between studies (*P* < 0.00001, *I*2 = 86%), and meta-analysis is performed by combining effect sizes with random-effects model. The results show that there is no significant difference in average maternal blood loss between the two groups (SMD = 0.10, 95% CI (−0.11, 0.32), *P*=0.35). According to the dosage of misoprostol, they are divided into ≥600 *μ*g group and <600 *μ*g group. In subgroup analysis, there is no statistical heterogeneity among studies in the misoprostol ≥600 *μ*g group (*P*=0.78, I2 = 0%), and the fixed-effect model is used for effect size analysis. The results show that there is no significant difference in average blood loss between misoprostol ≥600 *μ*g group and oxytocin group (SMD = 0.11, 95% CI (−0.04, 0.26), *P*=0.14). The results show that there is no significant difference in average maternal bleeding between misoprostol <600 *μ*g group and oxytocin group (SMD = 0.11, 95% CI (−0.04, 0.26), *P*=0.14). The results show that there is no significant difference in the mean maternal blood loss between the misoprostol <600 *μ*g group and the oxytocin group (SMD = 0.10, 95% CI (−0.21, 0.40), *P*=0.54).  Figure 3 displays the pooled standard mean difference of blood loss for 7 studies.

### 5.2. The Time of the Third Stage of Labor

The time of the third stage of labor is reported in five studies (2638 women). There is no statistical heterogeneity between studies (*P*=0.24, *I*2 = 28%). The results show that there is no significant difference in the time of the third stage of labor between the misoprostol group and the oxytocin group (SMD = 0, 95% CI (0.07, 0.08), *P*=0.95). According to the dosage of misoprostol, they are divided into ≥600 *μ*g group and <600 *μ*g group for subgroup analysis. There is no significant statistical heterogeneity among studies in the misoprostol ≥600 *μ*g group (*P*=0.15*P* = 0.15, *I*2 = 48%), and the fixed-effect model combined with effect size is used for analysis. The results show that there is no significant difference in the third stage of labor between the misoprostol ≥600 *μ*g group and the oxytocin group (SMD = 0.02, 95% CI (−0.07, 0.11), *P*=0.67). There is no statistical heterogeneity among studies in the misoprostol <600 *μ*g group (*P*=0.27, *I*2 = 19%). The results show that there is no significant difference between misoprostol <600 *μ*g group and oxytocin group in average blood loss (SMD = −0.04, 95% CI (−0.18, 0.10), *P*=0.60).  Figure 4 shows the pooled standard mean difference of the time of the third stage of labor for 5 studies.

### 5.3. The Incidence of Blood Transfusion

The incidence of blood transfusion is reported in nine studies (23,292 women) with no statistical heterogeneity between studies (*P*=0.45, *I*2 = 0%) and are analyzed using a fixed-effect model with effect size. The results show that there is no significant difference in the incidence of blood transfusion between the misoprostol group and oxytocin group (RR = 0.80, 95% CI (0.63, 1.02), *P*=0.07).  Figure 5 is the pooled rate of blood transfusion for 9 studies.

### 5.4. The Incidence of Shivering

The incidence of shivering is reported in nine studies [11–18, 22, 23] (23532 women) with statistical heterogeneity between studies (*P* < 0.00001, *I*2 = 93%) and is analyzed using a random-effects model combined with effect size. The results show that the incidence of maternal shivering in the misoprostol group is significantly higher than that in the oxytocin group, and the difference is statistically significant (RR = 2.61, 95% CI (1.79, 0.81), *P* < 0.00001). According to the dose of misoprostol, misoprostol is divided into ≥600 *μ*g group and <600 *μ*g group for subgroup analysis: there is systematic heterogeneity among all studies of misoprostol ≥600 *μ*g group (*P* < 0.00001, *I*2 = 94%), and random-effect model combined with effect size is used for analysis. The results show that the incidence of maternal shivering in misoprostol ≥600 *μ*g group is significantly higher than that in oxytocin group, the difference is statistically significant (RR = 2.61, 95% CI (1.79, 3.81), *P* < 0.00001). There is statistical heterogeneity among studies in the misoprostol <600 *μ*g group (*P* < 0.00001, *I*2 = 94%), and the random-effects model is used to combine effect size for analysis. The results show that the incidence of maternal shivering in misoprostol <600 *μ*g group is significantly higher than that in oxytocin group, the difference is statistically significant (RR = 3.99, 95% CI (1.65, 9.66), *P*=0.002) (Figure 6). However, sensitivity analysis results show that there is no directional change in the combined effect value after removing any one study, suggesting that the results of each subgroup are basically stable. Figure 6 shows the pooled rate of shivering for 9 studies.

### 5.5. The Incidence of Vomiting

The incidence of vomiting is reported in nine studies (22,463 women) with no statistical heterogeneity between studies (*P*=0.30, *I*2 = 16%) and is analyzed using a fixed-effect model with effect size. The results show that the incidence of maternal vomiting in misoprostol group is significantly higher than that in oxytocin group, and the difference is statistically significant (RR = 2.78, 95% CI (1.85, 4.18), *P* < 0.00001).  Figure 7 presents the pooled rate of vomiting for 9 studies.

The incidence of vomiting is used to analyze publication bias. It can be seen from Figure 8 that the symmetry of scattered point distribution of all studies is good, suggesting that there is no obvious publication bias in this index. Figure 8 displays the funnel plot for publication bias.

Severe postpartum bleeding needs to be considered for surgical treatment and can even lead to the removal of the uterus. Therefore, safe and effective drug selection is crucial in the prevention of postpartum bleeding. Causes of postpartum hemorrhage include uterine weakness, placental factors, soft birth canal injury, and coagulation disorders, among which weak uterine contractions hemorrhage is the most common cause of postpartum hemorrhage. At present, oxytocin has been used as a first-line drug to prevent postpartum hemorrhage in the guidelines of many countries and has been widely used in clinical practice. The mechanism of oxytocin is to activate the oxytocin receptor of the uterine smooth muscle, thereby enhancing the contractile tension of the uterine smooth muscle and improving the uterine contraction frequency, and finally achieving the purpose of hemostasis.

Oxytocin has the characteristics of quick action and few adverse reactions, and the half-life of the drug is only 3–4 min, the action time is relatively short, so it can be used many times. Chinese guidelines recommend that 10∼40 U be added into 500∼1000 mL liquid slowly or directly injected intramuscular with 10 U. However, the total dose should not exceed 60 U, which may cause adverse reactions such as water poisoning, coronary artery ischemia, and elevated blood pressure. Misoprostol is a prostaglandin E derivative, mainly used in obstetrics to prevent labor induction and postpartum bleeding. The dose is usually 200–600 *μ*g. In addition to oral administration, sublingual administration or anal penetration can also be adopted. Misoprostol has the advantages of convenient use, rapid absorption, and quick action and will not cause increased blood pressure or increase the load of the cardiovascular system.

A total of 13 RCTS involving 24,754 parturient women are included in this meta-analysis, including 12372 in experimental group and 12382 in control group. Meta-analysis shows that compared with the oxytocin group, there are no statistically significant differences in average blood loss, time to the third stage of labor, incidence of blood transfusion, and incidence of nausea in the misoprostol group. Misoprostol has the pharmacological activity of E-prostaglandin and can directly act on the uterus to produce rhythmic contraction, with the advantage of fast absorption and long acting time. Oral misoprostol can cause intense uterine contractions and reduce postpartum bleeding, thus reducing later surgical intervention due to bleeding. As can be seen from the results of this meta-analysis, misoprostol has the same effect as oxytocin in preventing postpartum hemorrhage, and its low price and relatively simple route of administration can be used as an alternative for emergency use in underdeveloped and remote areas where cold chain technology is lacking and sterile syringes are hard to obtain. However, the results of this meta-analysis also show that misoprostol had many adverse reactions. The frequency of adverse reactions is divided into common and occasional, corresponding to chills and vomiting, respectively. The incidence of maternal chills and vomiting in the misoprostol group is higher than that in the oxytocin group, because misoprostol could easily cause contraction of the intestinal smooth muscle. In addition, the drug can cross the blood-brain barrier through the transport of multidrug resistance-associated protein 4 (MRP4) and SLCO1B1, so its safety remains to be further discussed. In the process of use, the adverse reactions need to be closely observed and handled in time.

## 6. Conclusion

In conclusion, the effectiveness of misoprostol in preventing postpartum bleeding is similar to that of oxytocin, but the incidence of adverse reactions is high, and the occurrence of adverse reactions should be closely watched during the use. Due to the limitations of the included studies, this conclusion still needs to be further verified by multicenter, large-sample, and high-quality RCT in the future.

This study also has some limitations: (1) from the overall quality of the included literature, although the inclusion and exclusion criteria of this meta-analysis are strictly implemented, most of the included studies had a small sample size; (2) in different studies, the dosage of misoprostol and oxytocin is inconsistent, and the above factors may affect the accuracy of the conclusions of this meta-analysis.

## Figures and Tables

**Figure 1:** PRISMA flowchart for our literature search.

**Figure 2:** Risk of bias summary and risk of bias graph.

**Figure 3:** The pooled standard mean difference of blood loss for 7 studies.

**Figure 4:** The pooled standard mean difference of the time of the third stage of labor for 5 studies.

**Figure 5:** The pooled rate of blood transfusion for 9 studies.

**Figure 6:** The pooled rate of shivering for 9 studies.

**Figure 7:** The pooled rate of vomiting for 9 studies.

**Figure 8:** The funnel plot for publication bias.

**Table 1:** The baseline characteristics of included studies.

First author (year)	Country	Group	Age (mean ± SD), years	Sample size	Intervening measure	Outcomes
Atukunda (2014)	Uganda	Experimental group	29.3 ± 3.4	570	600 *μ*g misoprostol, sublingual	(2) (3) (4)
		Control group	29.7 ± 3.1	570	10 u oxytocin, intramuscular	
Bellad (2012)	Belgium	Experimental group	23.0 ± 3.1	321	400 *μ*g misoprostol, sublingual	(2) (3) (4) (5)
		Control group	22.8 ± 3.0	331	10 u oxytocin, i.v.	
Blum (2010)	Burkina Faso, Turkey, Egypt	Experimental group	25.0 ± 5.3	407	800 *μ*g misoprostol, sublingual	(3) (4) (5)
		Control group	25.0 ± 4.8	402	40 u oxytocin, i.v.	
Chaudhuri (2012)	India	Experimental group	22.07 ± 3.60	265	400 *μ*g misoprostol, sublingual	(1) (4)
		Control group	22.35 ± 2.97	265	10 u oxytocin, intramuscular	
Elbohoty (2016)	Egypt	Experimental group	27.9 ± 5.2	89	400 *μ*g misoprostol, sublingual	(1) (3) (4) (5)
		Control group	27.7 ± 5.5	86	10 u oxytocin, intramuscular	
Gülmezoglu (2001)	Argentina, China, Egypt, Ireland, Nigeria, South Africa, Switzerland, Thailand, Vietnam	Experimental group	26.5 ± 5.5	9264	600 *μ*g misoprostol, oral	(3) (4) (5)
		Control group	26.3 ± 5.4	9266	10 u oxytocin, i.v.	
Kundodyiwa (2001)	Zimbabwe	Experimental group	24.4 ± 5.6	243	400 *μ*g misoprostol, oral	(4) (5)
		Control group	23.8 ± 5.3	256	10 u oxytocin, i.v.	
Musa (2015)	Nigeria	Experimental group	29.60 ± 4.71	100	600 *μ*g misoprostol, oral	(1) (2) (4) (5)
		Control group	29.50 ± 4.37	100	10 u oxytocin, intramuscular	
Oboro (2003)	Nigeria	Experimental group	23.6 ± 5.2	247	600 *μ*g misoprostol, oral	(1) (2) (3) (5)
		Control group	23.9 ± 4.8	249	10 u oxytocin, i.v.	
Rajaei (2014)	Iran	Experimental group	25.86 ± 5.79	200	400 *μ*g misoprostol, oral	−1
		Control group	25.86 ± 5.79	200	10 u oxytocin, i.v.	
Singh (2009)	India	Experimental group	24.17 ± 2.57	75	400 *μ*g misoprostol, sublingual	(1) (3) (4) (5)
		Control group	24.27 ± 2.67	75	5 u oxytocin, i.v.	
Walley (2000)	Ghana	Experimental group	25.7 ± 5.0	203	400 *μ*g misoprostol, oral	(1) (3) (4) (5)
		Control group	26.1 ± 5.5	198	10 u oxytocin, intramuscular	
Çalişkan E (2003)	Turkey	Experimental group	24.4 ± 4.7	388	400 *μ*g misoprostol, oral	(1) (3) (4) (5)
		Control group	25.0 ± 5.1	384	10 u oxytocin, i.v.	

## Data Availability

The simulation experiment data used to support the findings of this study are available from the corresponding author upon request.
